The article "DEAF1 Is a Pellino1-interacting Protein Required for Interferon Production by Sendai Virus and Double-stranded RNA" was published in 2013. Journal: J Biol Chem.

# DEAF1 Is a Pellino1-interacting Protein Required for Interferon Production by Sendai Virus and Double-stranded RNA*[Fn FN2]

**DOI:** 10.1074/jbc.M113.479550

**Published:** 2013-07-11

**Authors:** Alban Ordureau, Karine Enesa, Sambit Nanda, Brice Le Francois, Mark Peggie, Alan Prescott, Paul R. Albert, Philip Cohen

**Affiliations:** From the ‡ MRC Protein Phosphorylation and Ubiquitylation Unit and; ¶ College of Life Sciences, Sir James Black Centre, University of Dundee, Dundee DD1 5EH, Scotland, United Kingdom and; the § Ottawa Hospital Research Institute (Neuroscience), Department of Cellular and Molecular Medicine, University of Ottawa, Ottawa K1H 8M5, Canada

**Keywords:** Cytokines/Interferon, Double-stranded RNA Viruses, Fibroblast, Interferon, Transcription Factors, DEAF1, IRF3, Pellino1, TBK1

## Abstract

Double-stranded (ds) RNA of viral origin, a ligand for Melanoma Differentiation-associated gene 5 (MDA5) and Toll-Like Receptor 3 (TLR3), induces the TANK-Binding Kinase 1 (TBK1)-dependent phosphorylation and activation of Interferon Regulatory Factor 3 (IRF3) and the E3 ubiquitin ligase Pellino1, which are required for interferon β (IFNβ) gene transcription. Here, we report that Pellino1 interacts with the transcription factor Deformed Epidermal Autoregulatory Factor 1 (DEAF1). The interaction is independent of the E3 ligase activity of Pellino1, but weakened by the phosphorylation of Pellino1. We show that DEAF1 binds to the IFNβ promoter and to IRF3 and IRF7, that it is required for the transcription of the IFNβ gene and IFNβ secretion in MEFs infected with Sendai virus or transfected with poly(I:C). DEAF1 is also needed for TLR3-dependent IFNβ production. Taken together, our results identify DEAF1 as a novel component of the signal transduction network by which dsRNA of viral origin stimulates IFNβ production.

## Teaser

**Background:** The E3 ligase Pellino1 is required for interferon (IFN) β production following infection with Sendai virus or poly(I:C).

**Results:** The transcription factor DEAF1 interacts with Pellino1 and, like Pellino1, is needed for transcription of the IFNβ gene.

**Conclusion:** DEAF1 is required for the production of IFNβ .

**Significance:** DEAF1 is a new signaling component required for IFNβ production.

## Introduction

Pellino was originally identified in *Drosophila melanogaster* as a protein that interacted with Pelle, the *Drosophila* orthologue of Interleukin-1 Receptor-associated Kinase (IRAK)^3^ (1), where it is required for the secretion of the anti-microbial peptide Drosomycin and innate immunity (2). In mammalian cells, there are three *peli* genes, which encode the three isoforms Pellino1, -2, and -3. The Pellinos are E3 ubiquitin ligases, but only display this catalytic activity when they are phosphorylated at particular serine and threonine residues. The phosphorylation and activation of Pellino1 is catalyzed *in vitro* by IRAK1, IRAK4 (3–5), TANK-binding kinase 1 (TBK1), and IKKϵ (6). We have reported that IRAK1 is the major protein kinase that activates the endogenous Pellino1 in IL-1-stimulated mouse embryonic fibroblasts (MEFs) or in HEK293 cells that stably express the interleukin 1 (IL-1) receptor, but TBK1 and/or IKKϵ appear to be the major Pellino1 activators in TNFα-stimulated MEFs or in the RAW264.7 macrophage cell line after stimulation with Toll-like Receptor (TLR) ligands (6, 7). In addition, prolonged stimulation of RAW264.7 cells or primary BMDM with the TLR4 agonist bacterial lipopolysaccharide (LPS) or the TLR3 agonist poly(I:C), a double-stranded (ds) RNA mimetic, greatly increases the expression of Pellino1 mRNA and protein (6, 8).

The article "DEAF1 Is a Pellino1-interacting Protein Required for Interferon Production by Sendai Virus and Double-stranded RNA" was published in 2013. Journal: J Biol Chem.

We recently generated knock-in mice in which wild type Pellino1 was replaced by an E3 ligase-deficient mutant (Pellino1[F397A]) and exploited them to demonstrate that Pellino1 is required for the production of IFNβ induced by the TLR3 ligand poly(I:C) in myeloid cells, or by infection with Sendai virus in mouse embryonic fibroblasts (MEFs) (9). It has been established that the effects of poly(I:C) and Sendai virus require the protein kinase TBK1, which catalyzes the phosphorylation of Interferon Regulatory Factor 3 (IRF3), causing it to translocate to the nucleus where it dimerizes and binds to the IFNβ promoter to stimulate transcription of the IFNβ gene (10). We showed that the poly(I:C)-stimulated interaction of IRF3 with the IFNβ gene promoter is reduced considerably in macrophages from the Pellino1[F397A] mice.

The first traces of IFNβ secreted in response to dsRNA activate a positive autocrine feedback activation loop that plays a critical role in generating the levels of IFNβ needed to combat viral infection. In this autocrine loop, IFNβ interacts with the type 1 interferon receptor, activating the JAK-STAT1/2 signaling network (11). This leads to the production of IRF7, a transcription factor that can also stimulates transcription of the IFNβ gene either by itself or as in a heterodimeric complex with IRF3. Moreover, IRF7 stimulates transcription of the genes encoding IFNα, which also activates the type 1 interferon receptor. Additionally, IFNβ stimulates transcription of the genes encoding RIG1 and MDA5 (12), which are cytosolic receptors that recognize the 5′-triphosphate of short dsRNA (RIG1) and longer dsRNAs of viral origin (MDA5). Once activated RIG1 and MDA5 interact with the mitochondrial anti-viral sensor (MAVS), which triggers the activation of a signaling network that also leads to the TBK1-catalyzed phosphorylation of IRF3.

The article "DEAF1 Is a Pellino1-interacting Protein Required for Interferon Production by Sendai Virus and Double-stranded RNA" was published in 2013. Journal: J Biol Chem.

To investigate how Pellino1 might act at the molecular level to stimulate IFNβ production, we carried out a yeast two-hybrid screen to identify interacting proteins. This led us to identify Deformed Epidermal Autoregulatory Factor 1 (DEAF1) (also called Nuclear DEAF1-Related (NUDR)) as a protein that binds to Pellino1. This observation was intriguing because, like Pellino1 (2), the transcription factor DEAF1 (13, 14) was originally identified as a gene required for the production of the anti-bacterial peptides Drosomycin and Metchnikowin in *D. melanogaster*. These observations led us to investigate whether DEAF1 might also be involved in regulating signaling networks of the mammalian innate immune system in which mammalian Pellino isoforms are involved. In this report, we show that, like Pellino1, mammalian DEAF1 is required for the transcription of the IFNβ gene induced by Sendai virus or poly(I:C).

## EXPERIMENTAL PROCEDURES

### 

#### 

##### Materials

Poly(I:C) was purchased from Invivogen, Lipofectamine^TM^ reagents from Invitrogen, benzonase (70746) from Novagen, Tofacitinib (CP690550) from Selleck Chemicals, and Ruxolitinib (INCB 1824) from Chemie-Tek. Rabbit and mouse secondary antibodies conjugated to horseradish peroxidase were from Pierce. Mouse interleukin-1α(IL-1α), anti-HA affinity matrix, anti-FLAG M2 antibody and affinity matrix, as well as anti-tubulin (T9026) were from Sigma-Aldrich. Phosphospecific antibodies that recognize p38α MAP kinase (p38α MAPK) phosphorylated at Thr-180 and Tyr-182 (9211), p105 phosphorylated at Ser-933 (4806), STAT1 phosphorylated at Tyr-701 ((9167), IRF3 phosphorylated at Ser-396 (clone# 4D4G) and antibodies recognizing all forms of IκBα (4814), TBK1 (3504), RIGI (3743), MDA5 (5321), and MAVS (3993) were purchased from Cell Signaling Technology. Anti-IRF3 (sc-15991X) was from Santa Cruz Biotechnology, and anti-HA was from Roche. Anti-GFP was made by the Division of Signal Transduction Therapy, MRC Protein Phosphorylation and Ubiquitylation Unit, University of Dundee, UK. Nanotrap GFP-binder affinity matrix was from ChromoTek. The DEAF1 antibody raised in rabbits has been described previously (15).

##### DNA Clones and Expression Vectors

The human Pellino1 construct for yeast two-hybrid screening pAS2.6 was created by cloning Pellino1 (GenBank^TM^ accession number AJ278859) from pSC-b Pellino1 (4) into the BamHI and Not1 sites of pAS2.6. The pCMVFLAG-1 Pellino1 for expression in mammalian cells was created as above, but cloning into pCMVFLAG-1. pEGFP-C1 Pellino1 encoding green fluorescent protein (GFP)-tagged Pellino1 was created by cloning Pellino1 from pSC-b Pellino1 into the BamHI site of EGFP-C1 (Clontech). Human DEAF1 (GenBank^TM^ accession number NM_021008.2) was amplified from IMAGE EST 6584290, cloned into pSC-b (Agilent), fully sequenced and subcloned into the BamHI sites of pCMVHA-1 or pEGFP-C1 (Clontech). Mouse DEAF1 (NCNI reference AAH46399.1) was amplified from IMAGE EST 5063995 using KOD Hot Start DNA polymerase (Merck). This was then cloned into the BamH1 and Not1 sites in pCMVFLAG-1. Mutants of mouse DEAF1, DEAF1[K251A], DEAF1[W253Q], DEAF1[K254A], DEAF1[H276S], DEAF1[R303T/K305T], were made by following the QuikChangeTM site-directed mutagenesis method (Stratagene), but using KOD Hot Start DNA Polymerase. pCMVFLAG-2 IRAK1 (GenBank^TM^ accession number AAC41949.1) was subcloned from pFBGST IRAK1 (4) and cloned into the Not1 site of pCMVFLAG-2. Human IRF3 (NCBI CAA91227.1) was amplified from IMAGE EST 5494536, subcloned into pSC-b, sequenced and then cloned into the Not1 site of pCMVHA-2. Human IRF7 (NCBI NP_001563) was amplified from IMAGE EST 5201404, subcloned into pSC-b, and cloned into the BamHI and Not1 site of pCMVHA-1. Human CREB was amplified with a 5′ HA-tag from IMAGE EST 3872792, cloned into pCR2.1 (Invitrogen) and subcloned into the EcoR1 and BamH1 sites in pCMV5. The IKKϵ constructs have been described elsewhere (16).

The article "DEAF1 Is a Pellino1-interacting Protein Required for Interferon Production by Sendai Virus and Double-stranded RNA" was published in 2013. Journal: J Biol Chem.

##### RNA Interference

siRNA transfection of HEK293-TLR3 cells was carried out using Lipofectamine^TM^ RNAiMAX Transfection Reagent. Conditions used for RNA transfection were as described by the manufacturer, and the amount of siRNA used is indicated in the figure legends. All siRNAs used were ON-TARGETplus SMARTpool (Dharmacon), resuspended according to the manufacturer's instructions. The siRNA pool targeting Human DEAF1 comprised four different oligonucleotide sequences (#1-CCAGAAGCUGCGUUGCCAA, #2-UAGAAGAGAUGGUCAACUC, #3-CGGGAGGCUAUGAGCGAGU, #4-GAUCAUGAGCGUCCGGUCU), the ON-TARGETplus Non-targeting Control Pool being used as negative control. After transfection, cells were left for 72 h and then stimulated with poly(I:C) for the times indicated in the figure legends.

##### Cell Culture and Cell Lysis

Bone marrow-derived macrophage (BMDMs) were differentiated for 7 days in RPMI medium (Roswell Park Memorial Institute) supplemented with 20% L929-conditioned medium as a source of M-CSF, 2 mm glutamine, 10% fetal bovine serum), 10 mm sodium pyruvate (Lonza), 0.1 mm 2-mercaptoethanol, 1 mm non-essential amino acids (Lonza), and the antibiotics penicillin and streptomycin (100 units/ml and 100 μg/ml, respectively). Embryonic fibroblasts from wild-type and DEAF1−/− mice (E15 embryos) were immortalized by infection with a lentivirus expressing the SV40 T antigen. The cell lines were established and genotyped as described (17). FLAG-tagged DEAF1 and DEAF1 mutants, subcloned into a retroviral expression vector (pBabe-puro vector), were used to obtain puromycin-resistant DEAF1-expressing MEFs. Each of the puromycin-resistant cell lines generated stably expressed DEAF1 or DEAF1 mutants as judged by immunoblotting with anti-FLAG antibodies. Human embryonic kidney (HEK) 293 cells that stably express the TLR3 receptor (a gift from Katherine Fitzgerald, University of Massachusetts), termed HEK-293-TLR3 cells, and HEK-293FT (Invitrogen) cells were cultured in DMEM (Dulbecco's-modified Eagle's medium) supplemented with 10% FBS, 2 mm glutamine, and the antibiotics penicillin and streptomycin (100 units/ml and 100 μg/ml, respectively). Cell transfections were performed by the Lipofectamine^TM^ 2000 method, as described by the manufacturer (Invitrogen). The culture medium was removed and after washing once with PBS, the cells were lysed with 1.0 ml of ice cold 50 mm Tris/HCl, pH 7.5, 1 mm EGTA, 1 mm EDTA, 1% (w/v) Nonidet P-40, 1 mm sodium orthovanadate, 10 mm sodium β-glycerophosphate, 50 mm NaF, 5 mm sodium pyrophosphate, 0.27 m sucrose, 1 mm benzamidine, 2 mm phenylmethanesulfonyl fluoride. The lysates were centrifuged at 16,000 × *g* at 4 °C for 15 min, and the supernatant, termed cell extract, was removed. Protein concentrations were determined using the Bradford method with bovine serum albumin as the standard.

The article "DEAF1 Is a Pellino1-interacting Protein Required for Interferon Production by Sendai Virus and Double-stranded RNA" was published in 2013. Journal: J Biol Chem.

##### Immunological Procedures

Cell extracts (5–10 μg) were denatured in SDS, resolved by electrophoresis on SDS/polyacrylamide gels, and electroblotted on to PVDF membranes. Membranes were blocked with 5% (w/v) skimmed milk in TBST (Tris-buffered saline with Tween 20: 50 mm Tris/HCl, pH 7.5, 0.15 m NaCl, and 0.1% (v/v) Tween 20) or with 5% (w/v) BSA in TBST. Detection of immuno-complexes was performed using horseradish peroxidase-conjugated secondary antibodies (Pierce) and an enhanced chemiluminescence reagent (GE Healthcare, Amersham Biosciences, UK). Native gel electrophoresis was carried out as described (18). For immunoprecipitations, anti-FLAG M2-agarose, anti-HA-agarose, or GFP-binder was utilized. Cell extracts (0.1 mg) were incubated for 1 h with 5 μl (packed volume) of coupled antibody or GFP-binder. Immune complexes were washed three times with cell lysis buffer supplemented with 0.25 m NaCl and resuspended with 10 mm Tris/HCl, pH 8.0. The immunoprecipitates were then centrifuged for 1 min at 2000 × *g* at 4 °C. The supernatant was discarded, and the immunoprecipitates denatured in SDS in the absence of any thiol to elute the bound proteins. The beads were recentrifuged for 1 min at 2000 × *g*, and the supernatants collected and subjected to SDS-PAGE.

The article "DEAF1 Is a Pellino1-interacting Protein Required for Interferon Production by Sendai Virus and Double-stranded RNA" was published in 2013. Journal: J Biol Chem.

##### Immunofluorescence

MEFs were fixed in 3.7% (v/v) formaldehyde, permeabilized with 0.1% (w/v) Triton X-100 in phosphate-buffered saline pH 7.4 and stained with anti-IRF3 antibody (Santa Cruz Biotechnology, sc15991) and Alexafluor 488-conjugated secondary antibodies (Invitrogen, A11055). The cells were mounted using ProLong antifade reagent with DAPI (Molecular Probes, P-36931), and the images were collected on a confocal microscope (LSM 510 META; Carl Zeiss MicroImaging) with 10 fields collected per coverslip. Images were quantified using the Volocity program (Perkin-Elmer). Nuclei were identified using the DAPI-stained channel while the mean intensity of IRF3 (green channel) in the nuclear region was measured. For each field the mean nuclear intensity was calculated, and this mean was used to calculate the overall mean nuclear intensity for each treatment.

##### Viral Infection

Sendai virus (SeV) (*Cantell Strain*) was supplied by Charles River Laboratories with a minimum HA titer of 4000 HA units/ml. MEFs from wild type and DEAF1−/− mice were seeded at 1 × 10^5^ in a 12-well plate. The following day, cells were infected using 100 HA units/ml in a serum free medium. Cells were incubated for 60 min at 37 °C with the virus in serum-free media. The serum-free media were then replaced by complete media, and the cells incubated at 37 °C for the times indicated in figure legends.

##### Quantitiative Real-time PCR

Total RNA was extracted from 1.2 × 10^6^ bone marrow-derived macrophages (BMDM) or HEK293-TLR3 cells using a Qiagen RNeasy kit following the manufacturer's instructions and quantitated by measuring the absorbance at 260 nm. 1 μg of total RNA was reverse transcribed into cDNA for 30 min at 42 °C using the qScript cDNA SuperMix from Quanta Biosciences. Then cDNA (50 ng) was incubated with primers (100 nm) in a total volume of 20 μl using the PerfeCT Syber Green Fast mix from Quanta Biosciences and the cDNA corresponding to the amplified mRNA was measured using the ΔΔ Cycle Threshold (CT) method and the constitutively expressed gene hypoxanthine phospho-ribosyl transferase or 18 S RNA as an internal control. The following primers were used in this study: Deaf1-F-5′-AGAATGAGCTGCCCACAACT-3′; Deaf1-R-5′-AGATCAAAGGTCAGTGCTCCAGA-3′; mHPRT-F-5′-GTTGGATACAGGCCAGACTTTGTTG-3′; mHPRT-R-5′-GAGGGTAGGCTGGCCTATAGGCT-3′; hIFNβ-F-5′-CTTTGCTATTTTCAGACAAGATTCA-3′; hIFNβ-R-5′-GCCAGGAGGTTCTCAACAAT-3′; mIFNβ-F-5′-GGAAAAGCAAGAGGAAAGATTGAC-3′; mIFNβ-R-5′-CCACCATCCAGGCGTAGC-3′; Pellino1-F-5′-CCTATGTCCCTCTGTGGCTTGG-3′; Pellino1-R-5′-GTGTGCGTACCATGAGGAAGTG-3′; mCXCL10-F-5′-CCTGCAGGATGATGGTCAAG-3′; mCXCL10-R-5′-GAATTCTTGCTTCGGCAGTT-3′; h18S-F-5′-GTAACCCGTTGAACCCCATT-3′; h18S-R-5′-CCATCCAATCGGTAGTAGCG-3′; mIFNα4-F-5′-ACCCACAGCCCAGAGAGTGACC-3′; mIFNα4-R-5′-AGGCCCTCTTGTTCCCGAGGT-3′; mIFNα6-F-5′-CAGGAGGTGGGGGTGCAGGA-3′; mIFNα6-R-5′-TCACTCGTCCTCACTCAGTCT-3′; mIL12p40-F-5′-TCATCAGGGACATCATCAAACC-3′; mIL12p40-R-5′-TGAGGGAGAAGTAGGAATGGG-3′; mIRF7-F-5′-GGGCTCCAAACCCCAAGCCC-3′; mIRF7-R-5′-CTGCGCTCGGTGAGAGCTGG-3′; Sendai virus Pgene-F-5′-GCATGGAGCCTGGCAGCTCA-3′; Sendai virus Pgene-R-5′-CGATTCAGCGGTGGGGACCG-3′; IRF1-F-5′-CCGAAGACCTTATGAAGCTCTTTG-3′; IRF1-R-5′-GCAAGTATCCCTTGCCATCG-3′; IL6-F-5′-TTCCATCCAGTTGCCTCTT-3′; Il6-R-5′-AGGTCTGTTGGGAGTGGTATC-3′; Iκbα-F-5′-ACACGTGTCTGCACCTAG-3′; Iκbα-R-5′-TCAGACGCTGGCCTCCAAAC-3′.

The article "DEAF1 Is a Pellino1-interacting Protein Required for Interferon Production by Sendai Virus and Double-stranded RNA" was published in 2013. Journal: J Biol Chem.

##### ELISA

The concentration of IFNβ released into the cell culture medium was determined by ELISA using a Verikine mouse IFNβ ELISA kit from PBL Interferon Source. The concentration of IFNβ in the cell culture medium was calculated using a standard curve established with known amounts of purified recombinant murine proteins.

##### Chromatin Immunoprecipitation

ChIP assays were performed using the ChIP-ITTM Express kit from Active Motif according to the supplier's instructions. Briefly, MEFs (4 × 10^6^ cells) from wild-type or DEAF1−/− mice were infected with Sendai virus, then cross-linked for 10 min with 1% formaldehyde at room temperature and the cells lysed. The chromatin was digested with DNase to an average size of about 300 bp, and the “sheared” chromatin incubated with shaking overnight at 4 °C with 2 μg of control IgG (Active Motif) or anti-IRF3 or anti-DEAF1 and 25 μl of protein G magnetic beads. The immune-precipitated DNA was purified with the MiniElute PCR purification kit from Qiagen, then incubated with primers (100 nm) in a total volume of 20 μl using the PerfeCT Syber Green Fast mix from Quanta Biosciences. The precipitated DNA was amplified and measured by real-time quantitative PCR. qPCR values were determined using the ΔΔ Cycle Threshold (CT) method using IgG and the constitutively expressed gene hypoxanthine phospho-ribosyl transferase as an internal control. The following primers were used: ChIP Ifnβ for 5′-GCC AGG AGC TTG AAT AAA ATG-3′; ChIP Ifnβ rev 5′-CTG TCA AAG GCT GCA GTG AG-3′.

## RESULTS

### 

#### 

##### DEAF1 Interacts with Pellino1

To identify proteins that interact with Pellino1, a yeast two hybrid screen was carried out using Pellino1 as bait. Approximately 4 × 10^6^ yeast colonies were screened from a human fetal brain cDNA library. One positive clone was identified as Pellino1 and another as Pellino3, suggesting that Pellino isoforms may be capable of homo- and hetero-dimerization, while a third was the E2 ubiquitin-conjugating enzyme Ubc13 (also called UBE2N) with which Pellino1 can form a productive complex to generate Lys63-linked polyubiquitin chains *in vitro* (4). A 4^th^ positive clone encoded SMAD6 (Similar to MAD (Mothers Against Pentaplegic), which has been reported to interact with the N-terminal region of Pellino1. The expression of SMAD6 and SMAD7 is induced by Transforming Growth factor β (TGFβ) and the interaction of MAD Homology 2 (MH2) domains of these SMADs with Pellino1 may modulate the TGFβ-stimulated inhibition of interleukin-1 (IL-1) and Toll-Like Receptor (TLR) signaling (19, 20). The identification of several known Pellino1-interacting proteins indicated that other positive clones detected during the screen also might encode proteins that were relevant to the function of Pellino1.

The article "DEAF1 Is a Pellino1-interacting Protein Required for Interferon Production by Sendai Virus and Double-stranded RNA" was published in 2013. Journal: J Biol Chem.

Another five positive clones identified in the screen encoded the C-terminal region of the transcription factor DEAF1, the smallest comprising residues 302–565. This finding was intriguing because Pellino1 and the *Drosophila* orthologue of DEAF1 are both required for the production of the anti-bacterial peptides Drosomycin and Metchnikowin in the fruit fly *D. melanogaster* (see Introduction), but were not considered to interact, since Pellino was reported to interact at the plasma membrane with Pelle, the *Drosophila* orthologue of IRAK, while DEAF1 functions in the nucleus. To investigate further whether Pellino1 and DEAF1 bind to one another, we co-expressed DNA vectors encoding hemagglutinin (HA)-tagged DEAF1 and either GFP-tagged Pellino1 (Fig. 1*A*) or FLAG-tagged Pellino1 (supplemental Fig. S1*A*) in HEK293FT cells. We found that the expressed HA-DEAF1 could be co-immunoprecipitated with GFP-Pellino1 using anti-GFP (Fig. 1*B*) or with FLAG-Pellino1 using anti-FLAG (supplemental Fig. S1*B*). Conversely, GFP-Pellino1 (Fig. 1*C*) or FLAG-Pellino1 (supplemental Fig. S1*C*) could both be immunoprecipitated with HA-DEAF1, using anti-HA. The results confirmed that these two proteins do indeed interact with one another.

**FIGURE 1.** **DEAF1 and Pellino1 interact in overexpression studies.** HEK293FT cells were transfected with DNA encoding HA-DEAF1 and/or GFP-Pellino1. After 36 h, the cells were lysed in buffer containing phosphatase inhibitors (see “Experimental Procedures”) plus 50 mm iodoacetamide. *A*, cell extracts (3 μg of protein) were denatured in SDS, subjected to SDS-PAGE, transferred on to a PVDF membrane, and immunoblotted (*IB*) with anti-HA and or anti-GFP to monitor the expression of the DEAF1 and Pellino1 fusion proteins. *B*, Pellino1 was immunoprecipitated (*IP*) from 0.1 mg of cell extract protein with the GFP antibody (GFP-Trap beads). The bound proteins were denatured in SDS, and immunoblotted with anti-HA and anti-GFP to detect DEAF1 and Pellino1, respectively. *C*, as in *B* except that DEAF1 was immunoprecipitated from 0.1 mg of cell lysate protein with an HA antibody. *D–F*, same as *A–C*, except that HA-DEAF1 was transfected with either wild-type (*WT*) or the F397A mutant (*F/A*) of Pellino1. *G* and *H*, same as *D*, *E* except that the cells were also transfected with FLAG-tagged wild-type (*WT*) IRAK1 or the catalytically inactive IRAK1[D358A] mutant (*D/A*). *I*, same as *A*, except that the cells were transfected with HA-DEAF1 and either wild-type FLAG-IKKϵ (WT) or the catalytically inactive FLAG-IKKϵ[D157A] mutant (*D/A*). The cell extracts were immunoblotted with anti-HA and anti-FLAG.

The article "DEAF1 Is a Pellino1-interacting Protein Required for Interferon Production by Sendai Virus and Double-stranded RNA" was published in 2013. Journal: J Biol Chem.

The interaction of Pellino1 with DEAF1 did not require the E3 ligase activity of Pellino1 since it was not decreased in cells transfected with DNA encoding the E3 ligase-inactive Pellino1[F397A] mutant (Fig. 1, *D–F*) (9). The co-transfection of DEAF1 and Pellino1[F397A] with a DNA vector encoding IRAK1 induced the phosphorylation and activation of Pellino[F397A], as shown by a decrease in its electrophoretic mobility (Fig. 1*G*). However, interestingly, the DEAF1 immunoprecipitates contained a much lower proportion of the phosphorylated, slower migrating form of Pellino1[F397A] (Fig. 1*H*) than was present in the cell extracts (Fig. 1*G*), indicating that the phosphorylation of Pellino1 weakens its interaction with DEAF1.

Interestingly, the co-transfection of DNA vectors encoding DEAF1 with wild-type IKKϵ, but not catalytically inactive IKKϵ, induced the phosphorylation of DEAF1, as shown by decreased electrophoretic mobility on SDS/polyacrylamide gels (Fig. 1*I*).

##### Reduced Production of IFNβ and IFNβ-dependent Genes in DEAF1−/− MEFs

We have reported that Pellino1 is required for the production of IFNβ in MEFs infected with Sendai virus (9). Since Pellino1 interacts with DEAF1 (Fig. 1 and supplemental Fig. S1), and Pellino and DEAF1 are both required in *Drosophila* for the production of anti-bacterial peptides (2, 13, 14), we investigated whether DEAF1 was required for the production of IFNβ.

The MEFs were infected with Sendai virus containing defective-interfering genomes, which strongly stimulate IFNβ production in these cells (21, 22). The dsRNA formed during the replication of these genomes is thought to stimulate IFNβ mainly by activating the MDA5-MAVS-TBK1-IRF3 pathway (23). The production of IFNβ mRNA (Fig. 2*A*) and IFNβ secretion (Fig. 2*B*) induced by infection with Sendai virus was reduced considerably in MEFs from DEAF1−/− mice compared with wild type controls. The mRNAs encoding IFNβ-dependent genes, such as IRF7 (Fig. 2*C*), IFNα4 (Fig. 2*D*), and IFNα6 (Fig. 2*E*), as well as CXCL10 (Fig. 2*F*) an established marker of viral infection, were also suppressed in DEAF1−/− MEFs. In contrast, the mRNAs encoding IκBα (Fig. 2*G*) or the pro-inflammatory cytokine IL-12p70 (Fig. 2*H*), which are controlled by the transcription factors NFκB (24) and IRF5 (25), respectively, were little affected. The expression of the Sendai virus nucleocapsid protein was not decreased in MEFs from the knock-in mice (Fig. 2*I*), indicating that the decreased production of IFNβ in DEAF1−/− MEFs was not due to the failure of the virus to infect the MEFs. Moreover, the IL-1-stimulated activation of p38α MAP kinase, the IKKβ-dependent phosphorylation of p105/NFκB1 or degradation of IκBα (supplemental Fig. S2*A*), or the IL-1-stimulated production of the mRNA encoding IRF1 (supplemental Fig. S2*B*) and CXCL10 (supplemental Fig. S2*C*) were unaffected in DEAF1−/− MEFs. Indeed, the production of IκBα mRNA (supplemental Fig. S2*D*) and IL-6 mRNA (supplemental Fig. S2*E*) in DEAF1−/− MEFs was increased slightly. Thus the reduced production of IFNs and IFN-regulated genes in DEAF1−/− MEFs was specific and did not result from a general loss in the transcription of many genes.

The article "DEAF1 Is a Pellino1-interacting Protein Required for Interferon Production by Sendai Virus and Double-stranded RNA" was published in 2013. Journal: J Biol Chem.

**FIGURE 2.** **The production of IFN**β **in Sendai virus infected MEFs is reduced in DEAF1−/− mice.** *A–I*, immortalized MEFs from wild type mice (*black bars*, *black circles* in *B*) or DEAF1−/− mice (*white bars*, *white squares* in *B*) were infected with Sendai virus (100 HA/ml) for the times indicated. Total RNA was extracted and analyzed by qRT-PCR to measure the mRNA encoding IFNβ, IRF7, IFNα4, IFNα6, CXCL10, IκBα, IL-12p40, and the Sendai virus Pgene. The results show fold increase in mRNA relative to the values measured in unstimulated MEFs (± S.D. for triplicate determinations). In *panel B*, the concentration of IFNβ in the culture medium was measured by ELISA. The results are shown ± S.D. for triplicate determinations. Similar results were obtained in four independent experiments using MEFs immortalized from two different wild type and two different DEAF1−/− mice.

##### DEAF1 Is Not Required for IFNβ-stimulated Gene Transcription

The production of IFNβ triggered by dsRNA of viral origin can be divided into two phases, an early phase in which IRF3 is activated and IFNβ gene transcription is initiated, and a second phase in which IFNβ activates the JAK-STAT1/2 signaling pathway, driving a positive feedback loop that gradually accelerates the rate of IFNβ production (see Introduction). To investigate whether DEAF1 exerted its effects at the second phase, we stimulated MEFs with IFNβ. These experiments revealed that the transcription of IFNβ-stimulated genes, was similar in MEFs from DEAF1−/− and DEAF1+/+ mice (Fig. 3, *A–D*). These genes included IRF7 (Fig. 3*D*), which is required for the positive feedback loop. The IFNβ-stimulated synthesis of MDA5 was also similar in MEFs from DEAF1−/− mice (Fig. 3*E*).

The article "DEAF1 Is a Pellino1-interacting Protein Required for Interferon Production by Sendai Virus and Double-stranded RNA" was published in 2013. Journal: J Biol Chem.

**FIGURE 3.** **IFNβ-stimulated signal transduction does not require DEAF1.** *A–D*, immortalized MEFs from wild type (*black bars*) and DEAF1−/− (*white bars*) mice were stimulated with 500 units/ml IFNβ for the times indicated. Total RNA was extracted and analyzed by qRT-PCR to measure the mRNA encoding CXCL10 (*A*), ISG15 (*B*), MX1 (*C*), and IRF7 (*D*). The results show fold increase in mRNA relative to the values measured in unstimulated MEFs (± S.D. for triplicate determinations). Similar results were obtained in two independent experiments. *E*, MEFs from wild type (DEAF1+/+) and DEAF1−/−) mice were stimulated with IFNβ as in *A–D*, and then lysed in the presence of phosphatase inhibitors. Aliquots of the cell extract (20 μg protein) were subjected to SDS-PAGE and, after transfer to PVDF membranes, immunoblotted with an antibody that recognizes STAT1 phosphorylated at Tyr-701 (p-STAT1) or that recognize MDA5 or TBK1.

##### Defective Recruitment of IRF3 to the IFNβ Promoter in MEFs from DEAF1−/− Mice

The results presented in the preceding section suggested that DEAF1 must be exerting its effects “upstream” of IFNβ secretion. Since DEAF1 is a transcription factor (13), we investigated whether it could bind to the IFNβ promoter and/or whether it affected the interaction of IRF3 with the IFNβ promoter. We showed that infection with Sendai virus enriched the association of IRF3 with IFNβ promoters in MEFs from wild type mice, which was maximal after 2 h, but this did not occur in MEFs from the DEAF1−/− mice (Fig. 4*A*). IFNβ promoters were not enriched if the anti-IRF3 was replaced by a control IgG (not shown). These ChIP experiments indicated that DEAF1 was required for the binding of IRF3 to the IFNβ promoter.

**FIGURE 4.** **IFNβ promoters associated with IRF3 are reduced in MEFs from DEAF1−/− mice.** *A*, MEFs from wild type mice (*black bars*) or DEAF1−/− mice (*white bars*) were infected with Sendai virus for the times indicated. The cells were lysed, and ChIP assays performed after immunoprecipitating IRF3 from the extracts with a specific anti-IRF3 antibody. The ordinate shows the fold enrichment of the IFNβ promoter in the anti-IRF3 immunoprecipitates compared with that measured after immunoprecipitation from uninfected cells (time = 0). The IFNβ promoter DNA was measured by qRT-PCR, as described in “Experimental Procedures.” The results are shown ± S.D. for triplicate determinations using MEFs from two different wild type and two different DEAF1−/− mice at each time point. Similar results were obtained in two independent experiments. *B*, experiment was carried out as in *A*, except that the ChIP assay was performed after immunoprecipitating DEAF1 from the extracts of MEFs from wild type mice (*black bars*) or from DEAF1−/− mice (*white bars*) with an anti-DEAF1 antibody.

The article "DEAF1 Is a Pellino1-interacting Protein Required for Interferon Production by Sendai Virus and Double-stranded RNA" was published in 2013. Journal: J Biol Chem.

Infection with Sendai virus also induced the association of the IFNβ promoter with DEAF1, as judged by its immunoprecipitation with anti-DEAF1 from the extracts of Sendai virus-infected wild type MEFs. This did not occur in extracts from uninfected cells or if the DEAF1 antibody was replaced by a control IgG. The association of DEAF1 with the IFNβ promoter followed similar kinetics to the association of IRF3 with the promoter (Fig. 4*B*). The DEAF1 antibody did not immunoprecipitate the IFNβ promoter from the extracts of Sendai virus-infected DEAF1−/− MEFs (Fig. 4*B*), indicating that the interaction was specific.

##### DEAF1 Stimulates IFNβ Gene Transcription

The finding that DEAF1 interacts with the IFNβ promoter and is required for IRF3 to interact with this promoter suggested that DEAF1 was likely to exert its effects by stimulating IFNβ gene transcription. We therefore stably transfected DEAF1−/− MEFs with either wild type or mutant forms of DEAF1 that are unable to stimulate gene transcription. These experiments showed that transfection with wild type mouse DEAF1 fully restored Sendai virus-induced IFNβ secretion to DEAF1−/− MEFs, but mutants of mouse DEAF1 lacking transcriptional activity could not (Fig. 5*A*). The mutations in the KDWK motif of the SAND domain (K251A, W253Q, K254A) prevent DEAF1 from binding to DNA (26), while the mutation of His-276 in the zinc binding motif to Ser also prevents DNA from binding to the SAND domain (27). The mutation of Arg-303 and Lys-305 to Thr, which prevents DEAF1 from entering the nucleus (28), has been shown to be transcriptionally inactive (26). Each mutant was expressed in MEFs at similar levels at similar levels to wild type DEAF1 (Fig. 5*B*). Thus the interaction of DEAF1 with DNA and its nuclear location are required to enhance the transcription of the IFNβ gene.

**FIGURE 5.** **DEAF1 transcriptional activity and nuclear localization is needed to stimulate IFNβ production.** *A*, immortalized MEFs from DEAF1−/− mice were stably reconstituted with either FLAG-tagged wild-type (*WT*) DEAF1, DEAF1[K251A], DEAF1[W253Q], DEAF1[K254A], DEAF1[H276S] and DEAF1[R303T/K305T]. These MEF cell lines, as well as the immortalized MEFs from wild type mice (+/+) and DEAF1−/− mice were infected with Sendai virus (SeV) (100 HA/ml) for the times indicated, and the concentration of IFNβ in the culture medium was measured by ELISA. The results are shown ± S.D. for triplicate determinations. *B*, the cell extract from *A* (25 μg protein) was denatured in SDS, subjected to SDS-PAGE, transferred to a nitrocellulose membrane, and immunoblotted (*IB*) with anti-FLAG to show the expression of the different DEAF1 mutants in the reconstituted MEFs.

The article "DEAF1 Is a Pellino1-interacting Protein Required for Interferon Production by Sendai Virus and Double-stranded RNA" was published in 2013. Journal: J Biol Chem.

It should be noted that K251, W253, K254, H276, R303, and K205 of mouse DEAF1 are equivalent to K250, W252, K253, H275, R302, and K204 of human DEAF1 (26–28) due to the insertion of an amino acid residue at position 89 in the mouse sequence.

##### DEAF1 Interacts with IRF3 and IRF7

Since DEAF1 and IRF3 appeared to bind to the same region of the IFNβ promoter, and DEAF1 is required for IRF3 to associate with the IFNβ promoter and to enhance IFNβ gene transcription, we wondered whether DEAF1 might interact with IRF3 directly. We therefore co-transfected DNA encoding GFP-tagged DEAF1 and HA-tagged IRF3 into 293FT cells (Fig. 6*A*). We found that GFP-DEAF1 was immunoprecipitated from the cell extracts with anti-HA (Fig. 6*B*) while, conversely, HA-IRF3 was immunoprecipitated with anti-GFP (Fig. 6*C*). Similar overexpression experiments revealed that DEAF1 could also interact with IRF7 (Fig. 6, *B* and *C*), which also binds to the IFNβ promoter where it may function alone or as a heterodimer with IRF3 (see Introduction). The interaction between DEAF1 and IRF3 or IRF7 was not affected by DNase treatment prior to immunoprecipitation (Fig. 6, *A–C*), indicating that the interactions were specific and not mediated indirectly by the binding of DNA to these transcription factors. CREB (cyclic AMP response element binding protein), another transcription factor, did not interact with DEAF1 (Fig. 6, *D–F*), again indicating that the interactions with IRF3/7 were specific.

**FIGURE 6.** **DEAF1 interacts with IRF3 and IRF7.** HEK293FT cells in 10-cm dishes were transfected with DNA (0.6 μg/ml) encoding GFP-DEAF1 and either HA-IRF3 or HA-IRF7. The cells were extracted in lysis buffer containing 50 mm iodoacetamide as in Fig. 1 and incubated for 2 h at 4 °C in the absence or presence of the DNase benzonase (50 units/ml). *A*, aliquots of the cell extract (3 μg protein) were subjected to SDS-PAGE and immunoblotted as in Fig. 1. *B*, IRF3 or IRF7 were immunoprecipitated from 0.1 mg of cell lysate protein with an HA antibody and the immunoprecipitates washed, denatured in SDS, and subjected to SDS-PAGE and immunoblotting as in *A. C*, as in *B* except that DEAF1 was immunoprecipitated using anti-GFP. *D–F*, as in *A–C* except that the cells were co-transfected with DNA encoding GFP-DEAF1 and HA-CREB.

The article "DEAF1 Is a Pellino1-interacting Protein Required for Interferon Production by Sendai Virus and Double-stranded RNA" was published in 2013. Journal: J Biol Chem.

##### The JAK-STAT1/2 Pathway Is Required for the Robust Phosphorylation and Dimerization of IRF3 in MEFs Infected with Sendai Virus or Transfected with Poly(I:C)

The results presented above indicated that DEAF1 exerted its effects by enhancing transcription of the gene encoding IFNβ. We were therefore initially surprised to observe that the phosphorylation and dimerization of IRF3 (Fig. 7, *A* and *B*, *panels P1* and *P2*) and its translocation to the nucleus (supplemental Fig. S3), which are earlier events in the signaling network, were also reduced considerably in DEAF1−/− MEFs, whether they were infected with Sendai virus (Fig. 7*A*) or transfected with poly(I:C) (Fig. 7*B*). However, even though the secretion of IFNβ was barely detectable 2 h post-infection/transfection, this was sufficient to induce near maximal phosphorylation of STAT1 at Tyr-701 (Fig. 7, *A* and *B*, *panel P4*). STAT1 phosphorylation was barely detectable in DEAF1−/− MEFs, presumably due to the much lower level of IFNβ secreted (Fig. 2). The phosphorylation of STAT1 was clearly catalyzed by the JAK kinases, since it was blocked by Ruxolitinib (Fig. 7, *C* and *D*, *panel P4*) or Tofacitinib (supplemental Fig. S4), which are potent, specific, and structurally unrelated JAK inhibitors (9). Importantly, the JAK inhibitors also suppressed the phosphorylation and dimerization of IRF3 (Fig. 7, *C* and *D*, *panels P1* and *P2*), indicating that the IFNβ-stimulated JAK-STAT pathway is required to detect robust activation of IRF3 2 h post-infection/transfection.

**FIGURE 7.** **The activation and synthesis of component of the interferon pathway in MEFs infected with Sendai virus or transfected with poly(I:C).** *A* and *B*, immortalized MEFs from wild type mice (DEAF1+/+) or DEAF1−/− mice were infected with Sendai virus (*SeV*) (100 HA units/ml) (*A*) or transfected with poly(I:C) (10 μg/ml) (*B*) for the times indicated. Cell lysates (30 μg protein) were denatured in SDS, subjected to SDS/PAGE, transferred to PVDF membranes and immunoblotted (*IB*) with the antibodies indicated. *Panel P2* shows a separate experiment in which SDS was excluded from the sample and native gel electrophoresis performed to separate the monomeric (*m*) and dimeric (*d*) forms of IRF3, which were then detected by immunoblotting. *C* and *D*, same as *A* and *B*, except that DEAF1+/+ MEFs were incubated for 1 h without (−) or with (+) 1 μm Ruxolitinib prior to infection with Sendai virus (*C*) or transfection with poly(I:C) (*D*).

The article "DEAF1 Is a Pellino1-interacting Protein Required for Interferon Production by Sendai Virus and Double-stranded RNA" was published in 2013. Journal: J Biol Chem.

A clue to the molecular mechanism underlying these results was obtained by studying the expression of MDA5 and RIG1, which are major cytosolic dsRNA receptors mediating the activation of IRF3 in Sendai virus-infected and poly(I:C)-transfected MEFs, respectively. The expression of MDA5 and RIG1 was strongly induced by Sendai virus or poly(I:C), was maximal within 2 h of infection/transfection, was not observed in DEAF1−/− MEFs (Fig. 7, *A* and *B*, *panels P5* and *P6*) and was prevented by Ruxolitinib and Tofacitinib (Fig. 7, *C* and *D*, *panels P5* and *P6* and supplemental Fig. S4). In contrast, the expression of MAVS, which operates “downstream” of MDA5 and RIG1 (29) was unaffected (Fig. 7, *panel P7*).

In summary, the results are consistent with DEAF1 exerting its effects at the level of IFNβ gene transcription, the consequent reduction in IFNβ secretion leading to a failure to activate the JAK-STAT pathway and to increase MDA5 and RIG1 expression to the level required for Sendai virus infection or poly(I:C) transfection to induce a sufficiently robust activation of IRF3 that it becomes detectable by immunoblotting.

##### DEAF1 Is Also Required for TLR3-dependent Production of Interferon β

To investigate whether DEAF1 was also required for TLR3-dependent IFNβ gene transcription, we initially used RNA interference (RNAi) to knock down the level of human DEAF1 mRNA (Fig. 8*A*). The reduction in DEAF1 expression greatly suppressed transcription of the IFNβ gene in HEK293-TLR3 cells (Fig. 8*B*) after stimulation with untransfected poly(I:C). In contrast, the production of mRNA encoding Pellino1 was unaffected (Fig. 8*C*).

**FIGURE 8.** **RNA interference of DEAF1 suppresses IFNβ mRNA production in poly(I:C)-stimulated HEK293-TLR3 cells.** HEK293 cells stably expressing the TLR3 receptor (termed HEK293-TLR3 cells) were transfected with “scrambled” siRNA (control) or with the indicated amounts of DEAF1-blocking siRNA. 72 h later, the cells were stimulated with poly(I:C) (50 μg/ml) for the times indicated, total RNA extracted and the mRNA encoding DEAF1 (*A*), IFNβ (*B*), and Pellino1 (*C*) was measured by qRT-PCR as described under “Experimental Procedures.” The results show relative mRNA levels (± S.D. for triplicate determinations) compared with the value of 1.0 measured in unstimulated control, HEK293-TLR3 cells. The experiment was performed in 12-well plates with three wells used for each condition. Similar results were obtained in two independent experiments.

DEAF1−/− mice are rarely born alive, and the few survivors are very small. Nevertheless, a few experiments with BMDM from DEAF1−/− mice were performed, which showed that the poly(I:C)-stimulated production of IFNβ mRNA (Fig. 9*A*) or CXCL10 (Fig. 9*B*) was reduced considerably compared with BMDM from wild-type mice. The reduction in IFNβ secretion (Fig. 9*C*) was similar to that observed in BMDM from mice expressing the E3 ligase-inactive Pellino1[F397A] mutant (Fig. 9*D*) (9).

The article "DEAF1 Is a Pellino1-interacting Protein Required for Interferon Production by Sendai Virus and Double-stranded RNA" was published in 2013. Journal: J Biol Chem.

**FIGURE 9.** **The poly(I:C)-stimulated production of IFNβ is impaired in BMDM from DEAF1−/− mice.** *A* and *B*, four wild type mice and three DEAF1−/− mice were used at each time point. BMDM from wild type (WT) (*black bars*) or DEAF1−/− mice (*white bars*) were stimulated for the times indicated with poly(I:C) (10 μg/ml) and, at each time point, the total RNA was extracted from the macrophages and the mRNA encoding IFNβ (*A*) and CXCL10 (*B*) was measured by qRT-PCR. The results show the fold increase in mRNA relative to the values measured in unstimulated, wild-type BMDMs (± S.D. for triplicate determinations). *C*, as in *A* and *B* except that, at each time point, the amount of IFNβ secreted into the cell culture medium from wild type BMDM (*black circles*) or DEAF1−/− BMDM (*white circles*) was measured by ELISA. *D*, same as *C*, except that BMDM from wild type (*WT*) mice (*black squares*) or Pellino1[F397A] mice (*white squares*) (9) were used.

## DISCUSSION

DEAF1 is known to play multiple roles *in vivo*. Through its role in controlling the production of serotonin, it has been linked to depression and suicide (15, 30, 31). It has also been linked to cancer (32, 33), type 1 diabetes (34), and neural tube defects (35). Here we identified DEAF1 as a Pellino1-interacting protein and showed that, like Pellino1, it positively regulates the binding of IRF3 to the IFNβ promoter, leading to the production of IFNβ mRNA, and hence IFNβ secretion, in response to Sendai virus or poly(I:C). We also show that DEAF1 is associated with the same region of the IFNβ promoter as IRF3, that it interacts with IRF3 and IRF7 and that DEAF1 mutants with impaired transcriptional activity fail to restore Sendai virus-induced IFNβ secretion to DEAF1−/− MEFs.

Full-length human DEAF1 displays 29% identity and 46% overall homology with *Drosophila* DEAF1. Human DEAF1 has an N-terminal region rich in alanine and acidic residues, which is absent in *Drosophila* DEAF1 or a shorter variant of mammalian DEAF1, termed Suppressin, in which Met-69 is used instead of Met-1 as the initiator methionine (28). However, all forms of DEAF1 share a DNA-binding SAND domain (named after **S**p100, **A**IRE-1, **N**ucP41/75, and **D**EAF1) comprising amino acid residues 193–273 in human DEAF1 (194–274 in mouse DEAF1). The SAND domain recognizes TTCG motifs in DNA through an α-helical surface patch containing the KDWK sequence that characterizes this domain (26, 36, 37). The TTCG sequences recognized by the SAND domain do not confer DEAF1-dependent transcriptional activation to the thymidine kinase promoter, suggesting that DEAF1 may activate transcription independently of promoter binding, perhaps by interaction with another protein(s) (28). One such protein is thought to be LIM-only protein 4 (LMO4). The mouse knock-outs of LMO4 and DEAF1 have similar phenotypes and are thought to cooperate with one another in the regulation of gene transcription (35).

The article "DEAF1 Is a Pellino1-interacting Protein Required for Interferon Production by Sendai Virus and Double-stranded RNA" was published in 2013. Journal: J Biol Chem.

The SAND domain is followed by a nuclear localization signal (NLS) (amino acid residues 301–316 of human DEAF1), a Nuclear Export Sequence (NES) (residues 454–476) (28) and a C-terminal Zinc Finger-Like region (residues 477–543), termed the MYND domain (after **My**eloid translocation protein 8, **N**ervy and **D**EAF1) (37). The MYND domain is a protein-protein interaction domain (27, 37) and the smallest Pellino1-interacting fragment detected in our yeast two-hybrid screen comprised amino acid residues 302–565 of DEAF1, which contains the NES and MYND domain. Interestingly, LMO4 interacts with amino acid residues 404–479 of DEAF1, which includes the NES. The interaction of DEAF1 with LMO4 was found to stimulate the nuclear accumulation of DEAF1 in overexpression studies, presumably because the NES was masked (38). In contrast to LMO4, we were unable to detect an interaction between Pellino1 and amino acid residues 404–479 of DEAF1.^4^

We found that DEAF1 became phosphorylated upon co-transfection with IKKϵ or TBK1 (Fig. 1*I*) and have identified five sites (Ser-140, Ser-156, Ser-197, Ser-213, and Ser-422) that are phosphorylated by IKKϵ *in vitro* or after co-transfection with IKKϵ.^5^ The phosphorylation of DEAF1 may facilitate nuclear entry and/or enhance the interaction of DEAF1 with IRF3, IRF7, and/or the IFNβ promoter. Ser-197 and Ser-213 are located within the SAND domain suggesting that their phosphorylation might enhance interaction with DNA. However, further work is needed to establish whether these sites are phosphorylated in the endogenous DEAF1 protein in response to Sendai virus or poly(I:C). These experiments are currently hampered by the low level of expression of DEAF1 in MEFs and myeloid cells and by lack of appropriate phosphospecific antibodies, and will also require the development of improved DEAF1 antibodies.

Taken together, our results suggest a model in which the TBK1/IKKϵ-catalyzed phosphorylation of IRF3, and perhaps DEAF1, induce their translocation to the nucleus where they bind to the IFNβ promoter to enhance IFNβ gene transcription. Since the DEAF1-Pellino1 interaction is weakened by the phosphorylation of Pellino1 (Fig. 1*H*), the phosphorylation-induced dissociation of DEAF1 from Pellino1 may permit DEAF1 to interact with LMO4 and translocate to the nucleus as the DEAF1-LMO4 complex.

The article "DEAF1 Is a Pellino1-interacting Protein Required for Interferon Production by Sendai Virus and Double-stranded RNA" was published in 2013. Journal: J Biol Chem.

The TBK1-catalyzed phosphorylation of DEAD-box helicase DDX3X has been reported to enable DDX3X to interact with the IFNβ promoter and to enhance IFNβ gene transcription (39, 40). Therefore, like many other genes, the transcription of the IFNβ gene seems to be controlled by the combinatorial actions of multiple transcription factors.

Sendai virus or poly(I:C) induced production of IFNβ is defective in MEFs and macrophages from knock-in mice expressing the E3 ligase inactive Pellino1[F397A] mutant (9). However, the interaction of DEAF1 with this mutant and wild type Pellino1 was similar, and DEAF1 did not undergo ubiquitylation when it was co-transfected with activated Pellino1. These observations suggest that the Pellino1-catalyzed ubiquitylation of another, as yet unidentified, protein may be needed to stimulate IFNβ gene transcription. However, it is also possible that the mutation of the RING domain disrupts another function of Pellino1 associated with either the RING domain itself or another domain of Pellino1 (41). Further studies are therefore needed to understand how and whether the E3 ligase activity of Pellino1 regulates IFNβ production.

## Footnotes

4 A. Ordureau, unpublished work.

5 A. Ordureau, results not shown.

## Footnotes

3 The abbreviations used are:

IRAK: interleukin-1 receptor-associated kinase
SeV: Sendai virus
DEAF: deformed epidermal autoregulatory factor
MEF: mouse embryonic fibroblast
TBK: TANK binding kinase.
